The article "lncRNA MSC-AS1/miRNA-429 Axis Mediates Growth and Metastasis of Nasopharyngeal Carcinoma via JAK1/STAT3 Signaling Pathway" was retracted in 2023. Reasons: signs of a paper mill; compromised peer review; unreliable results or conclusions.

# lncRNA MSC-AS1/miRNA-429 Axis Mediates Growth and Metastasis of Nasopharyngeal Carcinoma via JAK1/STAT3 Signaling Pathway

**DOI:** 10.1155/2022/1447207

**Published:** 2022-09-29

**Authors:** Ni Luo

**Affiliations:** Department of Otolaryngology, The Second Affiliated Hospital of Shandong University of Traditional Chinese Medicine, Jinan, Shandong 250001, China

## Abstract

**Objective:**

We attempted to clarify the effect of lncRNA MSC-AS1 on carcinogenic and development of nasopharyngeal carcinoma (NPC) and the related mechanisms.

**Methods:**

The levels of MSC-AS1 and miR-429 were estimated in NPC tissues and cells using qRT-PCR. Correlation analysis, dual-luciferase report, and RNA pull down assay assessed the action association of MSC-AS1 and miR-429. MTT, colony formation, cell wound scratch, and transwell assays were used to assess the proliferation, invasion, and migration of C666-1 cells. Metastasis-related protein expressions and activation of the JAK1/STAT3 pathway were confirmed by western blot and immunohistochemistry.

**Results:**

The expression of MSC-AS1 presented significant upregulation, and miR-429 expression was markedly downregulated in NPC tissues and cells. The level of MSC-AS1 had negative relation to the miR-429 level. Knockdown of MSC-AS1 suppressed the proliferation, invasion, and migration of C666-1 cells. On the contrary, overexpressing of MSC-AS1 exerts the opposite effects on C666-1 cell growth and migration. miR-429 was determined as functional downstream of MSC-AS1. The suppressive function of MSC-AS1 knockdown was predominately abolished by the miR-429 inhibitor. miR-429 was an antitumor gene inhibiting NPC growth and metastasis through JAK1/STAT3 pathway. In C666-1 cells, the elevated cell growth and migration induced by the miR-429 inhibitor were significantly reversed by si-JAK1 transfection.

**Conclusions:**

High expression of MSC-AS1 exerted a carcinogenic effect on NPC cell growth and metastasis by inhibiting miR-429 and activating the JAK1/STAT3 pathway.

## 1. Introduction

Nasopharynx-derived nasopharyngeal carcinoma (NPC) is a common form of all nasopharynx-related diseases [1]. Different from other head and neck cancers, NPC is an aggressive cancer, characterized by distal metastasis and rapid progression. It represents high morbidity in adolescents aged 15-24 years and elders aged from 65 to 79 years [2]. It is reported that over 0.12 million new cases are diagnosed with NPC in 2018 and 72,987 NPC-caused deaths occur around the world [3]. Although the incidence of NPC (0.7%) is relatively rare all over the world, NPC is prevalent in endemic regions, such as southern China and southeast Asia [4]. It is estimated that about 40% of new NPC cases of all NPC cases worldwide are diagnosed in China in 2018 [5]. Although the morbidity and mortality of NPC is declining in the past decade, effective treatment for NPC remains to be a challenge.

The article "lncRNA MSC-AS1/miRNA-429 Axis Mediates Growth and Metastasis of Nasopharyngeal Carcinoma via JAK1/STAT3 Signaling Pathway" was retracted in 2023. Reasons: signs of a paper mill; compromised peer review; unreliable results or conclusions.

Long noncoding RNA (lncRNA) is discovered as a subgroup of noncoding RNAs over 200 nucleotides long and exerts function in gene expression modulation via binding to miRNAs. A line of evidence has shown that lncRNAs exert key impacts on contributing to cancer progressions [6, 7]. LncRNA ATB presented elevation in renal cell carcinoma and promotes tumor cell growth [8]. LncRNA HOXA11-AS has been found to have a relation to breast cancer cell invasion and metastasis [9]. LncRNA H19 contributes to the invasion of glioma cells by targeting miRNA-675 [10]. LncRNAs have been suggested to be a promising target for cancer treatment.

MSC antisense RNA 1 (MSC-AS1), a novel lncRNA, exerts oncogenic functions in contributing to the development and progression of several cancers [11, 12]. Cao et al. demonstrated promoting the role of MSC-AS1 in hepatocellular carcinoma development by activating PGK1 [12]. MSC-AS1 is discovered to be a novel biomarker for laryngeal cancer diagnosis [13]. Additionally, MSC-AS1 presented a high level in NPC and exerted an oncogene in NPC by interacting with miR-524-5p and modulating NR4A2 [14]. Thus, MSC-AS1 may be a search focus in NPC.

Besides, lncRNAs present biological functions by sponging miRNAs. It is reported that MSC-AS1/miR-3924 exerts regulation in kidney renal clear cell tumor proliferation [15]. MSC-AS1 knockdown improved drug sensitivity by targeting miR-142 [16]. miR-429, belonging to the miR-200 family, participated in cancer development, metastasis, and progression [17]. It is reported that miR-429 is poorly expressed in NPC tissues and has a positive association with the prognosis of NPC patients. In addition, the downregulation of miR-429 is found in poorly differentiated NPC cells in comparison with well-differentiated ones [18]. The miR-429 expression had negative relation to MSC-AS1 in laryngeal cancer [13]. However, the interaction between miR-429 and MSC-AS1 in NPC remains elusive. Therefore, herein, we detected MSC-AS1 level in NPC tissues and cells and investigated the interactions of MSC-AS1/miR-429. The changes in NPC cell proliferation/migration/invasion were observed under MSC-AS1 knockdown. We attempted to explore the MSC-AS1 role in NPC. We anticipated our findings could provide novel insight into the NPC treatment modalities.

## 2. Methods

### 2.1. Patient and Tissue Sample Collection

The present study included 80 NPC patients aged from 25 to 69 years old who were admitted to the Second Affiliated Hospital of Shandong University of Traditional Chinese Medicine between January 2016 and March 2019. All the included patients were first diagnosed and treated in our hospital, without other malignant tumors and severe diseases. The tumor tissues and adjacent normal tissues of included patients were obtained under surgery and stored in liquid nitrogen for further analysis. In addition, patients with NPC were staged according to the American Joint Committee on Cancer (AJCC) staging system. The basic characteristics of patients were listed in Table 1. Informed consent was provided by patients or their parents. The Ethics Committee of the Second Affiliated Hospital of Shandong University of Traditional Chinese Medicine approved this study.

The article "lncRNA MSC-AS1/miRNA-429 Axis Mediates Growth and Metastasis of Nasopharyngeal Carcinoma via JAK1/STAT3 Signaling Pathway" was retracted in 2023. Reasons: signs of a paper mill; compromised peer review; unreliable results or conclusions.

### 2.2. Cell Culture

The normal nasopharyngeal epithelial cell line NP-69 and the NPC cell lines (HK-1, TW01, and C666-1) were purchased from the Chinese Academy of Sciences Cell bank (Shanghai, China). NP-69 cells were cultured in a keratinocyte-serum-free medium, and HK-1 cells were maintained in RPMI supplemented with 10% FBS and 1% double-resistance (Hyclone, Logan, UT, USA). C666-1 and TW01 cells were maintained in Dulbecco's modified eagle medium (DMEM) supplemented with 10% fetal bovine serum (FBS) and 1% double-resistance (Hyclone, Logan, UT, USA). All the cell lines were maintained at 37°C with 5% CO_2_ and 95% atmosphere.

### 2.3. Quantitative Reverse-Transcription Real-Time PCR (qRT-PCR) Analysis

Total RNA of tissue specimens and cells was isolated by Trizol solution. The purity and quality of RNA were determined by the ultraviolet absorption method. cDNA was reversely transcribed by using RT-PCR kit (Takara, Shiga, Japan) according to the manufacturer's instruction. PCR reaction was run under the ABI PRISM® 7500 system (Applied Biosystems, USA). The specific fragments of miR-429 and MSC-AS1 were amplified with the primers of miR-429 (forward: 5'-GGGGGTAATACTGTCTGGT-3' and reverse: 5'-TGCGTGTCGTGGAGTC-3'), MSC-AS1 (forward: 5'-AAGCAACAACTGTCTGGCCT-3' and reverse: 5'-TGATGCCAGCAAATTGGTGC-3'), and JAK1 (forward: 5'-ATTGGAGACTTCGGCCTGAC-3'; reverse: 5'-GGGTGTTGCTTCCCAGCATC-3'). The expression of miR-429 relative to U6 (forward: 5'-CTCGCTTCGGCAGCACA-3'; reverse: 5'-GCGAGCACAGAATTAATACGAC-3') and MSC-AS1, and JAK1 expression relative to GAPDH (forward: 5'-CAGCCTCAAGATCATCAGCA-3'; reverse: 5'-ATGATGTTCTGGAGAGCCCC-3') were analyzed based on the 2^−ΔΔCt^ method.

### 2.4. Cell Transfection

C666-1 cells (2 × 10^5^ cells/well) were seeded in a 6-well plate and cultured overnight to 70% confluence. MSC-AS1 gene fragment was amplified with Pfu DNA polymerase and inserted into pcDNA3.1 vector after being digested with Hind III and EcoR I. The reconstructed pcDNA-MSC-AS1 and pcDNA-NC vectors were transferred to cells through Lipofectamine 2000. In addition, si-MSC-AS1, si-NC, miR-429 inhibitor, miR-429 mimic, and miRNA-ctrl were purchased from Invitrogen (Shanghai, China).

The article "lncRNA MSC-AS1/miRNA-429 Axis Mediates Growth and Metastasis of Nasopharyngeal Carcinoma via JAK1/STAT3 Signaling Pathway" was retracted in 2023. Reasons: signs of a paper mill; compromised peer review; unreliable results or conclusions.

### 2.5. Western Blot

After being transfected for 48 h, cells were collected by centrifugation, followed by total protein extraction. The proteins were quantified by BCA (bicinchoninic acid) protein assay kit (Jianglaibio, Shanghai, China) and separated by 12% SDS-PAGE. Then, proteins were transferred to the PVDF membrane and blocked with 5% skim milk. The membranes were incubated with primary antibodies of MMP-2 monoclonal antibody (1 : 500, Invitrogen), MMP-9 polyclonal antibody (1 : 1000, Invitrogen), Cyclin D1 monoclonal antibody (1 : 200, Invitrogen), c-myc monoclonal antibody (1 : 200, Invitrogen), JAK1 monoclonal antibody (1 : 1000, Invitrogen), p-JAK1 polyclonal antibody (1 : 1000, Invitrogen), STAT3 monoclonal antibody (1 : 5000, Invitrogen), p-STAT3 polyclonal antibody (1 : 1000, Invitrogen), and GAPDH monoclonal antibody (1 : 1000, Invitrogen) at room temperature overnight, followed by incubation with the secondary antibody at 37°C for 90 min. Finally, proteins were detected with the ECL method under a multi-imager (Bio-Rap, Hercules, CA, USA).

### 2.6. MTT Assay

Cell proliferation was measured by using an MTT assay kit (Abcam, Cambridge, UK). Briefly, cells were seeded in a 96-well plate at a density of 1 × 10^3^ cells/well and cultured for 24 h. Then, cells were transfected with pcDNA-NC, pcDNA-MSC-AS1, si-MSC-AS1, si-NC, miRNA-ctrl, miR-429 inhibitor, and si-JAK1, respectively. Each experiment was performed in triplicate. After cells were cultured for 24, 48, and 72 h, respectively, MTT (0.1 mg) was added to each well and maintained for 4 h. Absorbance of cultures was obtained at 490 nm.

### 2.7. Dual-Luciferase Report Assay

The binding sites of MSC-AS1 and JAK1 for miR-429 were predicted by starBase 3.0 online tool (http://starbase.sysu.edu.cn/). The reconstructed pGL3-MSC-AS1-wild vector was obtained by inserting RNA sequence fragment containing the binding site of MSC-AS1. Meanwhile, pGL3-MSC-AS1-mut vector was constructed with mutant binding sequence. Then, C666-1 cells were seeded on a 96-well plate. When cultured to 70% confluence, cells were cotransfected with pGL3-MSC-AS1-wild/pGL3-MSC-AS1-mut and miR-429 mimic/miRNA-ctrl. After 48 h transfection, the luciferase signaling was detected. The target interaction between miR-429 and JAK1 was also detected as the method described above.

### 2.8. RNA Pull down

The relationship between MSC-AS1 and miR-429 was further determined by RNA pull down assay. Briefly, the biotin-labeled RNA probes (Bio-MSC-AS1 and Bio-NC) were incubated with cellular RNA extraction for 48 h. lncRNA-miRNA complex was extracted by combining with streptavidin beads. After eluting, the products were obtained for miR-429 level evaluation by qRT-PCR analysis.

The article "lncRNA MSC-AS1/miRNA-429 Axis Mediates Growth and Metastasis of Nasopharyngeal Carcinoma via JAK1/STAT3 Signaling Pathway" was retracted in 2023. Reasons: signs of a paper mill; compromised peer review; unreliable results or conclusions.

### 2.9. Colony Formation

After transfection for 48 h, cells were seeded in a 6-well plate at a density of 1000 cells per well and subsequently incubated in 2.5 ml medium for 14 days. After being washed, cells were fixed in methanol for 15 min at room temperature and stained with crystal violet. The colony formation was photographed under an inverted phase contrast microscope (Olympus Ckx53), and the colonies were counted with the application of ImageJ version 1.48 software.

### 2.10. Cell Wound Scratch Assay

Cells (5 × 10^5^ cells/well) were incubated in a 6-well plate. When cells were cultured to 90% confluence, the monolayer cells were scraped by the tip of 200 *μ*L pipette. After being washed with PBS, cells were maintained in serum-free medium for 24 h. The wound-healing area was photographed at 0 and 24 h of culture, and the wound-healing percentage was calculated according to the following formula:

(1) $$\begin{array}{c} \text{Wound healing percentage}=\frac{\text{ Area of wound}-\text{healing at }0\text{h}-\text{Area of wound}-\text{healing at }24\text{h}}{\text{Area of wound}-\text{healing at }0\text{h}}\times 100\%. \end{array}$$

### 2.11. Transwell Assay

After transfection, cells during the log phase were collected and resuspended. The upper chamber of transwell plate was pretreated with 200 *μ*L diluted Matrigel. Then, cells (5 × 10^4^ cells/ml) were seeded in the upper chamber, and the lower chamber was filled with 300 *μ*L RPMI-1640 media supplemented with 10% FBS. After cells were maintained at 37°C in 5% CO_2_ for 24 h, cells on the surface of the upper chambers were wiped off, and the remaining cells were fixed with 95% ethyl alcohol. Finally, cells were stained with 0.1% crystal violet and counted under a microscope.

### 2.12. Statistical Analysis

Statistical analysis was performed by SPSS17.0. Measurement data were expressed as mean ± standard deviation (SD). One-way ANOVA was applied to analyze the difference among multiple groups, and the pairwise differences were estimated by Tukey approach simultaneously. *p* < 0.05 was set as the significant threshold.

## 3. Results

### 3.1. The Levels of MSC-AS1 and miR-429 in NPC Tissues and Cells

The expressions of MSC-AS1 and miR-429 in NPC tissues and adjacent normal tissues were analyzed. MSC-AS1 presented higher expression in tumor tissues of NPC patients, compared with adjacent normal tissues (*p* < 0.001, Figure 1(a)). MSC-AS1 increased in tumor tissues in a grade-dependent manner (*p* < 0.001). All the included cases were divided into high (*n* = 45) and low MSC-AS1 groups (*n* = 35) based on MSC-AS1 median expression. A significant correlation between MSC-AS1 expression level and tumor stage (*p* = 0.004) was also analyzed in Table 1. Patients were followed up for about 5 years. High MSC-AS1 level had relation to poor prognosis (*p* < 0.001, Figure 1(b)). The expression of miR-429 was lower in tumor tissues than that in adjacent normal tissues and was significantly declined in advanced tumor tissues (stage III-IV) (all *p* < 0.001, Figure 1(c)). MiR-429 level had a negative association with MSC-AS1 level in NPC tissues (*p* = 0.021, Figure 1(d)).

The article "lncRNA MSC-AS1/miRNA-429 Axis Mediates Growth and Metastasis of Nasopharyngeal Carcinoma via JAK1/STAT3 Signaling Pathway" was retracted in 2023. Reasons: signs of a paper mill; compromised peer review; unreliable results or conclusions.

Additionally, we measured MSC-AS1 and miR-429 levels in three NPC cell lines and controls. MSC-AS1 was elevated in NPC cell lines relative to controls (all *p* < 0.05, Figure 1(e)). In contrast, miR-429 expression obviously decreased in NPC cells relative to controls (all *p* < 0.05, Figure 1(f)). Compared with the other NPC cell lines, C666-1 cells displayed a higher level of MSC-AS1 expression and lower miR-429 expression (all *p* < 0.05). Thus, the C666-1 cell line was selected for further assays.

### 3.2. MSC-AS1 Effects on the Proliferation, Migration and Invasion of C666-1 Cell

In order to analyze MSC-AS1 role in C666-1 cells, MSC-AS1 overexpressed, and knockdown cells were achieved by transfection with pcDNA-MSC-AS1, and si-MSC-AS1, respectively. QRT-PCR determined transfection efficiency. MSC-AS1 was remarkably accumulated in the pcDNA-MSC-AS1 group and declined in the si-MSC-AS1 group relative to pcDNA-NC, si-NC, and blank groups, respectively (all *p* < 0.01, Figure 2(a)). MSC-AS1 expression in pcDNA-NC, si-NC, and blank groups had not statistically different (*p* > 0.05). MTT revealed the increased cell viability in the pcDNA-MSC-AS1 group in a time-dependent manner but was obviously reduced in the si-MSC-AS1 group (all *p* < 0.01, Figure 2(b)). Similarly, C666-1 cells with MSC-AS1 overexpression showed obviously increased cell colonies in the pcDNA-MSC-AS1 group, while the colony formation ability of cells was remarkably reduced in MSC-AS1 silencing C666-1 cells (*p* < 0.001, Figure 2(c)). Cell wound scratch and transwell invasion assays evaluated the migration and invasion in C666-1 cells. Cells transfected with pcDNA-MSC-AS1 displayed prominently increased wound-healing ability, while si-MSC-AS1 transfected cells showed significantly declined wound-healing percentage at 24 h (*p* < 0.01, Figure 2(d)). Meanwhile, cell invasive ability was significantly elevated in the pcDNA-MSC-AS1 group but was markedly reduced under MSC-AS1 knockdown (all *p* < 0.01, Figure 2(e)).

The article "lncRNA MSC-AS1/miRNA-429 Axis Mediates Growth and Metastasis of Nasopharyngeal Carcinoma via JAK1/STAT3 Signaling Pathway" was retracted in 2023. Reasons: signs of a paper mill; compromised peer review; unreliable results or conclusions.

### 3.3. Relationship between lncRNA MSC-AS1 and miR-429

The binding site of MSC-AS1 and miR-429 were acquired from starBase 3.0 (Figure 3(a)). The pGL3-MSC-AS1-wild and pGL3-MSC-AS1-mut vectors were constructed by inserting MSC-AS1 binding sequences and mutant binding sequences into pGL3 vector, respectively. Double luciferase report assay showed that the luciferase signaling was markedly reduced in cells under pGL3-MSC-AS1-wild and miR-429 mimic cotransfection, compared to that in pGL3-MSC-AS1-wild and miRNA-ctrl cotransfection group (*p* < 0.01). However, there was no difference in luciferase activity in pGL3-MSC-AS1-mut inserted cells (*p* > 0.05, Figure 3(b)). RNA pull down exhibited accumulation of miR-429 in Bio-MSC-AS1 probe pulled down pellets, compared with controls (*p* < 0.001, Figure 3(c)). To further confirm the interaction between MSC-AS1 and miR-429, we detected miR-429 level in C666-1 cells after MSC-AS1 transfection. qRT-PCR illustrated that the miR-429 level was obviously reduced in MSC-AS1 overexpressed C666-1 cells, while significantly elevated after MSC-AS1 silencing (*p* < 0.001, Figure 3(d)). All these determined the binding of MSC-AS1 to miR-429.

### 3.4. The Carcinogenic Effect of MSC-AS1 on C666-1 Cells by Intervening miR-429 Expression

To detect whether MSC-AS1 exerted the carcinogenic effect on C666-1 cell malignancy by inhibiting miR-429 expression, the C666-1 cells received cotransfection with si-MSC-AS1 or miR-429 inhibitor. After transfection, qRT-PCR was used to examine miR-429 level. Results suggested that miR-429 expression increased in si-MSC-AS1+ miRNA-ctrl group, while it was obviously reduced in si-NC + miR-429 inhibitor (all *p* < 0.01). miR-429 inhibitor attenuated the increased miR-429 expression in MSC-AS1 silencing C666-1 cells (Figure 4(a)). MTT assessed the cell viability of C666-1 cells after transfection with si-MSC-AS1 and/or miR-429 inhibitor. Cell viability was notably declined in C666-1 cells transfected with MSC-AS1 inhibitor and pronouncedly elevated in miR-429 inhibitor, and MSC-AS1 inhibitor cotransfected C666-1 cells.. The suppressed cell viability in the si-MSC-AS1 + miRNA-ctrl group was partly abolished by transfected miR-429 inhibitor in C666-1 cells (*p* < 0.001, Figure 4(b)). The number of cell colonies decreased in the si-MSC-AS1 + miRNA-ctrl group and then reversely increased by miR-429 inhibitor (*p* < 0.001, Figure 4(c)). In addition, wound scratch and transwell assays evaluated the migration and invasion in C666-1 cells. Results showed that cell migration into the wound was obviously suppressed in MSC-AS1 knockdown C666-1 cells, which was rescued by miR-429 depletion (*p* < 0.001, Figure 4(d)). Similar findings were observed in transwell invasion assay, which suggested that the cell invasion ability was remarkably inhibited in cells transfected with si-MSC-AS1 + miRNA-ctrl but was obviously enhanced in the si-MSC-AS1 + miR-429 inhibitor group (all *p* < 0.05, Figure 4(e)). We did not discover a statistical difference in cell invasion in the si-NC + miRNA-ctrl and blank groups (*p* > 0.05). Thus, miR-429 depletion could reverse the declined C666-1 cell malignancy induced by MSC-AS1 silencing.

The article "lncRNA MSC-AS1/miRNA-429 Axis Mediates Growth and Metastasis of Nasopharyngeal Carcinoma via JAK1/STAT3 Signaling Pathway" was retracted in 2023. Reasons: signs of a paper mill; compromised peer review; unreliable results or conclusions.

### 3.5. miR-429 Knockdown Promotes the Proliferation, Migration and Invasion of C666-1 Cells through JAK1/STAT3 Pathway

To explore the miR-429 role in NPC and its relation to JAK1/STAT3 pathway, dual-luciferase report assays first determined the targeting of miR-429 to JAK1. Results showed that JAK1 was directly targeted by miR-429 (Figure 5(a)). Then, miR-429 inhibitor and si-JAK1 were transfected to C666-1 cells. qRT-PCR and western blot examined transfection efficiency. JAK1 expression at mRNA and protein level was markedly reduced after si-JAK1 transfection (all *p* < 0.01, Figures 5(b) and 5(c)). After transfection with si-JAK1, MTT and cell colony formation evaluated changes in C666-1 cell proliferation. Cell viability was significantly elevated in the miR-429 inhibitor + si-NC group, compared with controls, while it was rescued in cells transfected with miR-429 inhibitor + si-JAK1 (*p* < 0.001, Figure 5(d)). With a similar trend, the number of cell colonies increased after miR-429 depletion and then reversed after JAK1 silencing (*p* < 0.001, Figure 5(e)). To investigate the si-JAK1 influence on cell migration and invasion, we conducted cell wound scratch and transwell experiments. As shown in Figure 5(f), the wound-healing speed was higher under miR-429 downregulation and then rescued by JAK1 knockdown (*p* < 0.001, Figure 5(f)). Transwell assay revealed that knockdown of miR-429 by miRNA inhibitor transfection significantly elevated the cell invasion, compared with controls (all *p* < 0.01). Conversely, cotransfection with si-JAK1 efficiently inhibited miR-429 knockdown-induced cell invasion (*p* < 0.01, Figure 5(g)).

### 3.6. MSC-AS1 Targeting miR-429 Accelerates NPC Progression via the JAK1/STAT3 Pathway

To clarify the involvement of the JAK1/STAT3 pathway in MSC-AS1-induced NPC progression, immunohistochemistry measured the levels of p-JAK1 and p-STAT3 in NPC tumor tissues and controls. The p-JAK1 and p-STAT3 levels were accumulated in tumor tissues, compared with normal controls (Figure 6(a)). JAK1/STAT3 pathway activation in C666-1 cells was evaluated under si-MSC-AS1, miR-429 inhibitor, and si-JAK1 transfection. Western blot demonstrated that MSC-AS1 knockdown significantly suppressed p-JAK1 and p-STAT3 levels in C666-1 cells. On the contrary, miR-429 downregulation markedly reversed the reduced phosphorylation of JAK1 and STAT3 mediated by MSC-AS1 knockdown, while further adding si-JAK1 transfection remained the declined phosphorylation levels of JAK1 and STAT3 in C666-1 cells induced by MSC-AS1 knockdown in si-MSC-AS1 + miRNA-ctrl group (all *p* < 0.05, Figures 6(b)–6(d)).

The article "lncRNA MSC-AS1/miRNA-429 Axis Mediates Growth and Metastasis of Nasopharyngeal Carcinoma via JAK1/STAT3 Signaling Pathway" was retracted in 2023. Reasons: signs of a paper mill; compromised peer review; unreliable results or conclusions.

We further examined whether JAK1/STAT3 pathway was involved in the tumor growth and migration regulated by MSC-AS1. Results revealed that MMP2, MMP9, Cyclin D1, and c-myc expressions significantly decreased by MSC-AS1 knockdown, and the inhibition was obviously abolished by cotransfection with miR-429 inhibitor (all *p* < 0.001). MMP2, MMP9, Cyclin D1, and c-myc expressions in si-MSC-AS1 + miRNA-ctrl group were comparable to that in si-MSC-AS1 + miR-429 inhibitor + si-JAK1 group (*p* > 0.05, Figures 6(e) and 6(f)). Therefore, JAK1/STAT3 pathway was involved in the progression and development of NPC mediated by MSC-AS1 and miR-429 interaction.

## 4. Discussion

NPC is a kind of endemic disease with high prevalence in southern China. Despite advances in treatment efficacy, 30% of NPC patients were troubled with metastasis and recurrence of NPC [19]. Efforts have been made in novel therapeutic target discovery and new therapy development. Plenty of recent evidences have shown that MSC-AS1, as a lncRNA, plays a carcinogenic role in serval cancers [12, 20]. miR-429 involved in epithelial-mesenchymal transition, is a biomarker for the diagnosis, progression, and prognosis of cancers [17]. However, the role of the MSC-AS1/miR-429 axis in NPC has not been thoroughly investigated. In our study, we determined the expression level of MSC-AS1 in NPC tissues and cells. The effect of MSC-AS1 knockdown on the proliferation, migration, and invasion of NPC cells was investigated, and its related mechanism was further explored. We aimed to provide the clue for novel NPC therapeutic target discovery.

Our data showed that MSC-AS1 was significantly overexpressed in NPC tissues, compared with adjacent normal tissues, which was also determined in NPC cell lines. A similar expression profile of MSC-AS1 was observed in hepatocellular carcinoma (HCC) tissues and cells [12]. Our study also suggested that high MSC-AS1 expression was significantly correlated with poor prognosis of NPC patients. Besides, our data showed that MSC-AS1 knockdown by siRNA transfection significantly inhibited the proliferation, migration, and invasion of NPC cells. Li et al. also found that MSC-AS1 knockdown significantly suppressed cell proliferation and promoted cell apoptosis of glioma [20]. Collectively, the oncogenic role of MSC-AS1 in NPC was confirmed in the present study.

lncRNA plays a key role in regulating gene expression by binding to their target miRNAs. It is reported that MSC-AS1/miR-29b-3p plays a regulatory role in the proliferation and apoptosis of pancreatic ductal adenocarcinoma cells [11]. In our study, we found that MSC-AS1 inhibited miR-429 expression by binding to the complementary sequences and affecting the biofunction of miR-429 in NPC.

The article "lncRNA MSC-AS1/miRNA-429 Axis Mediates Growth and Metastasis of Nasopharyngeal Carcinoma via JAK1/STAT3 Signaling Pathway" was retracted in 2023. Reasons: signs of a paper mill; compromised peer review; unreliable results or conclusions.

MiR-429 family members have been reported to exert tumor suppressor function in multiple tumors [21, 22]. Previous evidences showed that miR-429 could promote cell apoptosis of nephroblastoma [22] and was predicted to be a biomarker correlated with poor prognosis of NPC. In this paper, we found that the expression of miR-429 was negatively correlated with MSC-AS1 expression in NPC tissues. The interactions between miR-429 and MSC-AS1 were validated by dual-luciferase report and RNA pull down assay. Moreover, inhibition of miR-429 expression could weaken the tumor suppressor effect of MSC-AS1 knockdown in NPC cells. Thus, we concluded that high expression of MSC-AS1 played an oncogenic role in NPC by suppressing the biofunction of miR-429.

Besides, signal transducer and activator of transcription 3 (STAT3) is a transcription factor that plays a pleiotropic role in cell processes such as immune response, cell growth, and cell vitality. Janus kinase 1 (JAK1), responsible for phosphorylating STAT3, is another critical member of the JAK1/STAT3 signaling pathway. JAK1/STAT3 pathway is activated in many malignant tumors and plays a critical role in promoting cancer initiation [23, 24]. A previous study showed that JAK1/STAT3 pathway was activated in colorectal cancer cells, accompanied by the increased phosphorylation level of JAK1 and STAT3 [25]. In our study, the phosphorylation level of JAK1 and STAT3 was obviously higher in PNC tissues than in the adjacent normal tissues. MiR-429 inhibited the proliferation, migration, and invasion of PNC cells via the JAK1/STAT3 signaling pathway. The phosphorylation of JAK1 and STAT3 was significantly reduced after MSC-AS1 knockdown, which was abolished by miR-429 inhibition. These results indicated that high expression of MSC-AS1 activated the JAK1/STAT3 pathway by mediating miR-429.

Furthermore, it is reported that STAT3 is correlated with tumorigenesis and tumor metastasis by regulating Cyclin D1, c-myc, MMP-2, and MMP-9 [26, 27]. Our study revealed that knockdown of MSC-AS1 suppressed the JAK1/STAT3 pathway, paralleled by significantly downregulated cell cycle-related factors (Cyclin D1 and c-myc), and metastasis-related proteins (MMP-2 and MMP-9). Therefore, high expression of MSC-AS1 contributed to the growth and metastasis of NPC by activating the JAK1/STAT3 signaling pathway.

The article "lncRNA MSC-AS1/miRNA-429 Axis Mediates Growth and Metastasis of Nasopharyngeal Carcinoma via JAK1/STAT3 Signaling Pathway" was retracted in 2023. Reasons: signs of a paper mill; compromised peer review; unreliable results or conclusions.

In conclusion, miR-429 was a direct functional target of MSC-AS1. High expression of MSC-AS1 promoted proliferation, invasion, and migration of PHC cells by activating the JAK1/STAT3 signaling pathway by suppressing miR-429. MSC-AS1/miR-429/STAT3 axis may be a promising target for NPC treatment.

## Figures and Tables

**Figure 1:** MSC-AS1 and miR-429 levels in NPC tumor tissues and cells. (a) MSC-AS1 expression was detected in tumor and adjacent normal tissues from 80 NPC patients by qRT-PCR analysis. The expression of MSC-AS1 was significantly higher in tumor tissues than in normal ones. (b) Patients were classified into high MSC-AS1 expression and low expression groups based on the median. The survival curve showed that high MSC-AS1 expression was negatively correlated with survival time. (c) The expression of miR-429 was measured in NPC tumor and adjacent normal tissues by qRT-PCR analysis. MiR-429 expression was obviously lower in tumor tissues, compared with normal controls. (d) Pearson analysis was conducted to analyze the correlation between the expression of MSC-AS1 and miR-429. The result showed that MSC-AS1 and miR-429 expression exhibited a negative relationship in NPC tissues. (e) The expression level of MSC-AS1 was detected in NPC cell lines (C666-1, HK-1, and TW01) and normal NP-69 cells. MSC-AS1 expression was significantly increased in NPC cell lines, compared with NP-69. ^∗^*p* < 0.05, ^∗∗^*p* < 0.01, and ^∗∗∗^*p* < 0.001. (f) The expression of miR-429 was detected in NPC cell lines (C666-1, HK-1, and TW01) and normal NP-69 cells by qRT-PCR analysis. miR-429 expression was markedly declined in NPC cell lines. ^∗^*p* < 0.05, ^∗∗^*p* < 0.01, and ^∗∗∗^*p* < 0.001.

**Figure 2:** Effect of abnormal MSC-AS1 effect on C666-1 cell proliferation, migration, and invasion. (a) The transfection efficiency was tested by qRT-PCR analysis. The expression of MSC-AS1 was remarkably accumulated in the pcDNA-MSC-AS1 group and significantly declined in the si-MSC-AS1 group compared with controls. ^∗^*p* < 0.05, ^∗∗^*p* < 0.01, and ^∗∗∗^*p* < 0.001. (b) The cell viability changes disturbed by MSC-AS1 dysregulation were detected by MTT assay. Cell viability was significantly reduced in the si-MSC-AS1 group. ^∗^*p* < 0.05, ^∗∗^*p* < 0.01, and ^∗∗∗^*p* < 0.001. (c) cell proliferation was observed by cell colony formation assay. The colony formation ability was significantly elevated in the pcDNA-MSC-AS1 group and obviously decreased in the si-MSC-AS1 group. NS: no significant difference; ^∗∗∗^*p* < 0.001. Cell wound scratch assay (d) and transwell invasion assay (e) were performed to observe the changes in migration and invasion of C666-1 cells induced by MSC-AS1 deregulation. The cell migration and invasion were all significantly enhanced in the pcDNA-MSC-AS1 group and reduced in the si-MSC-AS1 group. NS: no significant difference; ^∗∗^*p* < 0.01; ^∗∗∗^*p* < 0.001.

The article "lncRNA MSC-AS1/miRNA-429 Axis Mediates Growth and Metastasis of Nasopharyngeal Carcinoma via JAK1/STAT3 Signaling Pathway" was retracted in 2023. Reasons: signs of a paper mill; compromised peer review; unreliable results or conclusions.

**Figure 3:** The relationship between MSC-AS1 and miR-429. (a) The binding site between MSC-AS1 and miR-429 was predicted by starBase, and the mutant binding sequence was designed. (b) Double luciferase report assay was performed to validate the target interaction between MSC-AS1 and miR-429. Results determined that miR-429 was the direct target for MSC-AS1. ^∗∗^*p* < 0.01. (c) RNA pull down analysis was conducted to further validate the interaction between MSC-AS1 and miR-429. miR-429 could be pulled down by Bio-MSC-AS1-pellets complex. NS: no significant difference; ^∗∗∗^*p* < 0.001. (d) The interaction between MSC-AS1 and miR-429 was detected by qRT-PCR analysis after perturbed MSC-AS1 expression. Results showed that the expression of miR-429 was obviously reduced in MSC-AS1 overexpression cells, while significantly elevated after MSC-AS1 silence. NS: no significant difference; ^∗∗∗^*p* < 0.001.

**Figure 4:** The carcinogenic effect of MSC-AS1 on C666-1 cells is disturbed by intervening miR-429 expression. (a) After the C666-1 cells were cotransfected with si-MSC-AS1 and miR-429 inhibitor, the expression of miR-429 was measured by qRT-PCR analysis. The increased miR-429 expression induced by MSC-AS1 silence was repressed by the miR-429 inhibitor. NS: no significant difference; ^∗∗^*p* < 0.01; ^∗∗∗^*p* < 0.001. (b) Cell viability after cotransfected with si-MSC-AS1 and miR-429 inhibitor was estimated by MTT assay. Cell viability was significantly declined by MSC-AS1 expression inhibition, which was abolished by cotransfected with miR-429 inhibitor. ^∗∗∗^*p* < 0.001, compared with controls. (c) Colony formation assay was performed to analyze the cell proliferation. The number of cell colonies was significantly decreased after MSC-AS1 knockdown and was reversely increased after cotransfected with miRNA-429 inhibitor. NS: no significant difference; ^∗∗∗^*p* < 0.001. (d) Cell migration ability was observed by wound scratch. Cell migration was obviously suppressed in MSC-AS1 knockdown cells and was reversed by cotransfection with miRNA-429 inhibitor. NS: no significant difference; ^∗∗∗^*p* < 0.001. (e) Cell invasion ability was evaluated by transwell assay. Cell invasion ability was remarkably inhibited in cells transfected with si- MSC-AS1 + miRNA-ctrl but was obviously enhanced in the si-MSC-AS1 + miR-429 inhibitor group. NS: no significant difference; ^∗^*p* < 0.05; ^∗∗∗^*p* < 0.001.

The article "lncRNA MSC-AS1/miRNA-429 Axis Mediates Growth and Metastasis of Nasopharyngeal Carcinoma via JAK1/STAT3 Signaling Pathway" was retracted in 2023. Reasons: signs of a paper mill; compromised peer review; unreliable results or conclusions.

**Figure 5:** miR-429 knockdown promotes the proliferation, migration, and invasion of C666-1 cells through JAK1/STAT3 pathway. (a) The binding site between miR-429 and JAK1 was predicted by starBase. The mutant binding sequence was designed for dual-luciferase report assay. The luciferase signaling was significantly declined in JAK1 wild group transfected with miR-429 mimic. ^∗∗^*p* < 0.01, compared with miRNA-ctrl group. After being transfected with si-JAK1, the mRNA expression (b) and protein expression (c) of JAK1 was detected by RT-PCR analysis and western blot analysis, respectively. Results showed that JAK1 expression significantly declined, suggesting the transcription efficiency was high. NS: no significant difference; ^∗∗^*p* < 0.01; ^∗∗∗^*p* < 0.001. (d) Cell colony formation assay was performed to evaluate cell validity. Cell vitality was significantly elevated after being cultured for 24, 48, and 72 h in the miR-429 inhibitor + si-NC group and reversed after being transfected with si-JAK1. ^∗∗∗^*p* < 0.001. (e) Cell colony formation assay showed that the number of cell colonies was significantly increased in miR-429 knockdown cells and obviously reversed after cotransfected with si-JAK1. NS: no significant difference; ^∗∗∗^*p* < 0.001. Cell wound scratch (f) and transwell assay (g) were conducted to further investigate the effect of si-JAK1 on cell migration and invasion. The migration and invasion ability of C666-1 cells were significantly elevated in the miR-429 inhibitor + si-NC group. NS: no significant difference; ^∗∗^*p* < 0.01; ^∗∗∗^*p* < 0.001.

**Figure 6:** MSC-AS1 sponging miR-429 accelerates NPC progression via the JAK1/STAT3 pathway. (a) The expression of p-JAK1 and p-STAT3 in NPC and adjacent normal tissues were observed by immunohistochemical analysis. Results showed that expression levels of p-JAK1 and p-STAT3 were accumulated in tumor tissues. Scale bar = 100 *μ*m (b); after being transfected with miR-429 inhibitor, si-MSC-AS1, and si-JAK1, western blot analysis was performed to evaluate the changes in p-JAK1 and p-STAT3 expression. The expression of p-JAK1 (c) and p-STAT3 (d) significantly declined in si-MSC-AS1 + miRNA-ctrl and si-MSC-AS1 + miR-429 inhibitor + si-JAK1 group. NS: no significant difference, ^∗^*p* < 0.05, ^∗∗^*p* < 0.01, and ^∗∗∗^*p* < 0.001. (e) The tumor growth and metastasis-related proteins were detected by western blot analysis. (f) The expression of MMP2, MMP9, Cyclin D1, and c-myc was significantly reduced in si-MSC-AS1 + miRNA-ctrl and si-MSC-AS1 + miR-429 inhibitor + si-JAK1 group. NS: no significant difference; ^∗∗∗^*p* < 0.001.

The article "lncRNA MSC-AS1/miRNA-429 Axis Mediates Growth and Metastasis of Nasopharyngeal Carcinoma via JAK1/STAT3 Signaling Pathway" was retracted in 2023. Reasons: signs of a paper mill; compromised peer review; unreliable results or conclusions.

**Table 1:** Relationship between expression of MSC-AS1 and variables in NPC patients.

Variables		*N*	lncRNA MSC-AS1 level		*P* value
			Low (35)	High (45)	
Gender	Male	50	20	30	0.146
	Female	30	14	16	

Age	≤45	32	18	14	0.854
	>45	48	26	22	

Tumor stage	I-II	30	10	20	0.004
	III-IV	50	4	46	

N: number; *p* < 0.05 is considered significant.

## Data Availability

All data generated or analyzed during this study are included in this published article.

## Abbreviations

NPC: Nasopharyngeal carcinoma
lncRNA: Long noncoding RNA
MSC-AS1: MSC antisense RNA 1
qRT-PCR: Quantitative reverse-transcription real-time PCR
BCA: Bicinchoninic acid
SD: Standard deviation
MTT: 3-(4,5-dimethylthiazol-2-yl)-2,5-diphenyltetrazolium bromide
STAT3: Signal transducer and activator of transcription 3
JAK1: Janus kinase 1.
